This article has been retracted.

# Effective Ways for College Students' Mental Health Education Based on Music Therapy

**DOI:** 10.1155/2022/3031064

**Published:** 2022-01-11

**Authors:** Juncai Hou

**Affiliations:** School of Music, Xinxiang University, Xinxiang, Henan 453000, China

## Abstract

Music therapy plays a very important role in college students' mental health education. As a marginal subject, music therapy combines music, medicine, and psychology, which is beneficial to alleviate students' bad emotions and psychological problems and help college students form a sound personality. In the process of teaching in colleges and universities, it is necessary to choose teaching methods that are closer to students' real life so as to promote the healthy development of college students' psychology. From the relevant investigation and analysis, college students are interested in learning music, which provides an effective basis for college students to use music to treat psychological problems. Good policies, conditions, and a broad mass base are conducive to the application of music therapy in college mental health education. The application of music therapy in the field of college students' mental health also broadens the application field of music. This paper analyzes the application of music therapy in college students' mental health education and probes into the effective ways for college students' mental health education.

## 1. Introduction

Music therapy is a new and interdisciplinary subject. It is not only an art, but also a science, a process of interpersonal interaction, or a form of therapy. As a new discipline, it is still in the process of continuous development [1]. Making use of the advantage that music is easy to be accepted by college students, through individual music psychotherapy and group music counseling activities, we can help college students to alleviate bad emotions, solve psychological conflicts, and promote personality improvement, which is required by the current situation of mental health education in colleges and universities [2]. In the process of teaching in colleges and universities, we need to choose teaching methods that are more close to students' real life to promote the development of college students' mental health. From the relevant investigation and analysis, college students are interested in learning music, which provides an effective basis for college students to use music to treat psychological problems [3]. Music therapy is a systematic intervention process. In this process, therapists use various forms of music experience as well as the treatment relationship developed in the process of treatment, as the driving force of the treatment, to help the treatment object achieve the goal of health [4]. Music therapy can let college students vent their emotions in the appropriate environment and atmosphere and then guide them correctly to get out of the haze and welcome the sunshine [5].

Music therapy is a new and interdisciplinary subject. It is not only an art but also a science, a process of interpersonal interaction, and a form of treatment [6]. As a new subject, it is still in the process of continuous development. From the current situation of college students' mental health education, many colleges and universities do not attach great importance to this subject, which leads to many college students' immature psychological development and weak pressure resistance ability, which have adverse effects on the development of college students' physical and mental health [7]. Under the current situation, college students are facing increasing pressure, and the pressure comes from many aspects. College students are more sensitive to society, and their psychological control ability is weak, which is easy to produce a series of psychological problems. In the process of treatment, psychological counselors often use music therapy to help students come out of the past psychological shadow, reface the past memories, and help them learn to live with a more positive and better attitude [8]. Research on the application of music therapy in college students' mental health education can not only promote the innovation of college students' mental health education but also improve the education effect, which is of great significance to the development of college students' physical and mental health [9]. This paper analyzes the application of music therapy in college students' mental health education and probes into the effective ways of college students' mental health education.

As a new psychotherapy method, music therapy has its unique advantages. Its rich treatment methods can effectively meet the diversified mental health needs of college students. This paper creatively analyzes the application of music therapy in college students' mental health education and probes into the effective ways of college students' mental health education. In the process of college students' mental health education, music therapy plays an irreplaceable role.

## 2. The Role of Music Therapy in College Students' Mental Health Education

### 2.1. Helps to Improve Mood

In view of the effective role of music in emotional regulation, the new and potential music therapy has become one of the effective means of mental health education for college students. Through the light and pleasant music therapy technology, college students can effectively dispel their bad emotions and reconstruct themselves to develop good social adaptation. Music therapy is actually to use music to regulate people's physiological mechanisms and treat people's biological effects. With the rhythm of music, people's parasympathetic nervous system will be stimulated continuously. When everyone is stimulated by the external environment, people will feel happy or sad. The function of the parasympathetic nervous system is to relieve the tension and excitement of the human mechanism, so that people can enter a relaxed state. Music is the emotional language of people, which adjusts people's emotions to the maximum through physiological and psychological ways, guides people to send their inner thoughts to music, and finally plays the role in evacuation, depression, and empathy. Emotion is the first motive system of human beings, which determines the cognitive direction and personality development direction of human beings. Music has a great influence on people's emotions. It is worth noting that college students are in the mature stage of physical and mental development and gradually enter society, so they may have doubts about many social problems or phenomena, even show psychological barriers, which are all manifestations of mental loss, and need mental rehabilitation in mental health education.

Music therapists use music's great influence on emotions to improve people's emotions and finally change people's cognition. The purpose of psychological education activities is to guide college students to establish correct emotional values [10]. According to the basic and complex features of music, the overall features of music are identified. See Figure 1 for the specific structure.

In the evaluation of rhythm, the choice of a good rhythm will have a positive impact on the effect of the music, so it is assigned according to Table 1.

Spectrum flatness describes the flatness of the power spectrum and is the range of the boundary function:

(1) $$\begin{array}{c} K_{i}=\frac{t*\text{sqrt}\left(Ne\right)+\alpha }{L+\beta }. \end{array}$$

If the interval difference between two adjacent notes is greater than the octave, it will be recorded as *X*_*R*_:

(2) $$\begin{array}{c} X_{R}\left(k+1\right)=A_{R}X_{R}\left(k\right). \end{array}$$

With the increase of iteration times, the audience's favorite degree will occupy a more important proportion. That is,

(3) $$\begin{array}{c} V\left(k+1\right)=v\left(k\right)+e\left(k\right). \end{array}$$

Functional imaging shows that music, as a special sensory experience, has the ability to stimulate people's special strong emotions, and the emotions stimulated by the music can regulate the activities of the brain limbic system and paralimbic system structures, which play a key role in the formation, generation, maintenance, regulation, and retention of emotions. In the development of mental health education, music therapy is introduced, and under the alternation of rhythm and melody, people's emotional experience is mobilized, and psychological barriers and psychological problems are relieved. It can be seen that music therapy has a positive effect on strengthening students' emotional experience when applied to college students' mental health education. The purpose of psychological education activities is to guide college students to establish correct emotional values. It is helpful for college students to overcome psychological obstacles. It is helpful to cultivate students' ability of unity and cooperation, such as some abovementioned activities in music therapy, and also helps in analysis of students' psychological obstacles. It is conducive to cultivating college students' innovative thinking. There is an obvious division of labor in the left and right brains of humans, of which the right brain is for creative thinking. Influenced by the beauty of music, the painful emotional experience and life experience of humans are gradually transformed into a tragic aesthetic experience, which is sublimated and eventually become a rare spiritual wealth in life, and their personality is maturing accordingly. In music therapy, other forms, such as role-playing and music performance, can create specific situations for students. While enjoying fun, students know how to use music to express their emotions and get a successful experience.

### 2.2. Helps to Improve the Ability to Communicate with Others

In psychological counseling cases, college students are often caught in various bad emotions. Therefore, for college students, how to identify, manage, and control their emotions and strive to be the master of emotions are very important. It is easy for the cooperative spirit in music activities to migrate to real life, which helps most students who are pessimistic and self-enclosed to open their hearts, promote their ability to communicate and understand with others, and build a good relationship with others while knowing themselves correctly. For college students whose psychological state is not yet stable, the rapid development of science and technology, the fierce competition in society, the impact of ideas, the increasing employment pressure, economic pressure, and many uncertain factors have directly affected the physical and mental health of college students. The most common and greatest function of music in life is to reduce stress and relax one's mind and body.

For music, it is not good to keep the pitch rising or falling. Use the following formula to evaluate the overall outline of a piece of music:

(4) $$\begin{array}{c} G^{m}={\left[G_{1}^{T},G_{2}^{T},\ldots ,G_{k}^{T}\right]}^{T}. \end{array}$$

For the chorus, the pitch changes relatively quickly, such as the formula

(5) $$\begin{array}{c} A^{T}G=\sum_{i}A_{i}^{T}G_{i}. \end{array}$$

For music, it is not good to keep the pitch rising or falling. Use the following formula to evaluate the overall outline of a piece of music:

(6) $$\begin{array}{c} G_{i}^{\left(m\right)}=\left\{\begin{array}{c} I_{m},\;i=m,\\ 0_{m},\;i\neq m. \end{array}\right. \end{array}$$

For the chorus, the pitch changes relatively quickly, such as the formula

(7) $$\begin{array}{c} S_{1}=R_{1}=\left[G^{1},G^{2},\ldots ,G^{k}\right]. \end{array}$$

In the process of music therapy, we need to choose music-related activities, such as music creation, impromptu singing, and music games, but most people just think that music therapy is listening to music and relaxing. In the process of music therapy, there are mainly two forms: individual and collective. Under the guidance of music therapists, individuals train through music audition and singing, so as to build a harmonious relationship between teachers and students and improve students' language expression ability and emotional expression ability. The linear regression curve is calculated according to the stepwise multiple linear regression equation, as shown in Figure 2.

In music therapy, we should focus on visitors, be good at using rich music theories and excellent works at home and abroad as well as modern music production techniques, consider factors suitable for the personality, interest, IQ, and EQ of the parties, and choose appropriate music and music therapy methods to implement music therapy. Another advantage of music as a nonverbal communication lies in the fuzziness of its communication. Words are often discontinuous and limited. Music can express indescribable feelings of words and can also support individual feelings. Sociologists tell us that just as we create music, music also shapes us, and music promotes and corrects various social interactions. In the stage of higher education, it is an important period for college students to shape their personality, and music can play a positive role in cultivating human sentiment and promoting the realization of emotional training. In the process of college students' mental health education, if teachers can effectively apply music therapy, they can improve the effectiveness of education and teaching and promote the healthy development of college students' minds and bodies.

## 3. Music Therapy in Contemporary College Students' Mental Health Education

The excessive publicity of news media and excessive marketing of enterprises make the effect of music therapy appear the problem of excessive publicity, which makes the majority of college students form the wrong cognition in music therapy, and there is bias in music therapy. The college music therapy curriculum system is a social system engineering, in that schools, families, and society should work together to increase publicity. We should vigorously carry out campus music culture activities, make use of the strong educational radiation advantage of the Internet, provide music therapy, download all kinds of music or online audiovisuals, and build a healthy and civilized network culture with the characteristics of the times and meeting the needs of college students. Colleges and universities need to pay attention to the propaganda work of music therapy, carry out lectures and public elective courses in colleges and universities, use campus bulletin boards, campus networks, and other channels to guide students to correctly understand music therapy, feel the benefits of music therapy, and mobilize students' enthusiasm to participate in music therapy. Optimizing teachers' individual quality includes optimizing teachers' moral quality, knowledge quality, ability quality, and psychological quality. Music therapy teachers should have excellent music professional skills, and at the same time, they should master the related knowledge of psychological quality, education, and medicine [11]. Music and music therapists are no longer the important means of music therapy at this level. Music therapists make students aware of the causes of tension and the consequences in the process of exploring their interpersonal relationships by means of music activities selected for students. College music therapists need not only rich music knowledge but also professional knowledge of psychology, medicine, and pedagogy. Due to the limitations of the college environment, music therapists need to really love students and enhance their affinity. The teacher is the executor of the means in the process of music therapy. Therefore, the psychological quality of the executor plays an important role in the effect of music therapy [12]. Emotion plays an undeniably important role in the formation of human personality and cognition. At the same time, music can affect our emotions from some aspects. Therefore, we can use music therapy to stabilize students' emotions and make their values, world outlook, and outlook on life develop in a positive direction. In the process of music therapy, music therapists need to create a quieter, more harmonious, and more comfortable treatment environment for college students so that students can be in a relaxed and comfortable state in the process of treatment.

Music teachers in colleges and universities have very strong music abilities. Music teachers should not only have the basic knowledge of music but also have the knowledge of pedagogy and psychology. With the help of the training of psychological counselors, they can improve their comprehensive quality. Colleges and universities can also encourage medical psychological counselors to participate in the study of music and cultivate more people to engage with music therapy. People of different ages may not have the same language, but the beautiful melody of music can interact. Through music therapy, young and old relatives can narrow the generation gap caused by age differences. The use of music can not only build a more relaxed and comfortable consulting environment, but also build a harmonious relationship between music therapy counselors and students, using audition and games to build effective music therapy activities to promote the mental health development of college students. The application of music therapy in college students' mental health education mainly starts from the intervention at the support level, reeducation level, and reconstruction level, adopts various music therapy intervention methods, establishes the psychological connection with students through music, and stimulates the psychological, emotional, and cognitive experience through music so as to achieve the goal of mental health education.

## 4. Conclusions

Music therapy for college students' mental health problems is simple, effective, convenient, and fast, but we should pay attention to some details in the treatment. As a new method of psychotherapy, music therapy has its unique advantages. Its rich treatment methods can effectively meet the diversified needs of college students for mental health. It is necessary for colleges and universities to actively carry out college students' mental health education activities through effective teaching strategies so as to guide students to keep a good mood, more actively deal with difficulties and frustrations, establish a correct outlook on life and values, and realize their own life value. In the process of college students' mental health education, music therapy plays an irreplaceable role. Music therapy can effectively intervene in the mental health of college students, promote their physical and mental health, improve their psychological quality, guide them to form healthy personality, and cultivate their sentiment. The promotion of music therapy to the field of college students' mental health education effectively expands the channels of college students' mental health education and further promotes the innovation and development of college students' mental health education.

## Figures and Tables

**Figure 1:** Composition of the music form.

**Figure 2:** The relationship between the actual value and the calculated value of stepwise linear regression.

**Table 1:** Rhythm weight data.

Number of notes	Rhythm weight
Greater than 30	0.8
Greater than 20 and less than 30	0.6
Less than 30	0.4

## Data Availability

The data used to support the findings of this study are included within the article.
